This article has been retracted.

# Study on the Effect of Oral Administration of Bacteriophages in Charles Foster Rats With Special Reference to Immunological and Adverse Effects

**DOI:** 10.3389/fphar.2021.615445

**Published:** 2021-04-12

**Authors:** Mayank Gangwar, Sonam Rastogi, Digvijay Singh, Alka Shukla, Neeraj Dhameja, Deepak Kumar, Rajesh Kumar, Gopal Nath

**Affiliations:** ^1^ Viral Research and Diagnostic Laboratory, Faculty of Medicine, Department of Microbiology, Institute of Medical Sciences, Banaras Hindu University, Varanasi, India; ^2^ Department of Pathology, Institute of Medical Sciences, Banaras Hindu University, Varanasi, India

**Keywords:** oral, adverse effect, cytokines, *Klebsiella pneumoniae*, bacteriophage therapy

## Abstract

Numerous pre-clinical and clinical studies have recently demonstrated the significant role of phage therapy in treating multidrug-resistant bacterial infections. However, only a few researchers have focused on monitoring the phage-mediated adverse reactions during phage therapy. Besides adverse reactions, immunological response after short- and long-term oral administration of bacteriophages is also lacking. In this study, we administered the bacteriophages orally against *Klebsiella pneumoniae* XDR strain in dosages of 10^15^ PFU/ml and a 10^20^ PFU/ml (still higher) to Charles Foster rats as a single dose (in acute toxicity study) and daily dosage for 28 days (in sub-acute toxicity study). One milliliter suspension of bacteriophages was administered through the oral gavage feeding tube. No adverse effect was observed in any of the experimental as well as in the control animals.Further, an insignificant change in food and water intake and body weight was observed throughout the study period compared with the control group rats. On the 28th day of phage administration, blood was collected to estimate hematological, biochemical, and cytokines parameters. The data suggested no difference in the hematological, biochemical, and cytokine profile compared to the control group. No significant change in any of the treatment groups could be observed on the gross and histopathological examinations. The cytokines estimated, interleukin-1 beta (IL-1β), IL-4, IL-6, and INF-gamma, were found within the normal range during the experiment. The results suggested no adverse effect, including the severe detrimental impact on oral administration of high (10^15^ PFU/ml) and very high dose (10^20^ PFU/ml) of the bacteriophages cocktail. The high and long-term oral administration of bacteriophages did not induce noticeable immunological response as well.

## Introduction

The emergence of multi-drug resistant bacteria has forced humankind to look for alternatives to antibiotics. In the recent time alternative approaches have focused on the development of different biologicals that includes 1) passive immunization with pathogen-specific immunoglobulin preparations, 2) induction of a pathogen-specific memory response through vaccination, 3) immune-stimulatory agents leading to potentiation of host immune response facilitating clearance of the extracellular and intracellular infecting microbe, and 4) elimination of pathogenic bacteria by using lytic bacteriophages (Zumla et al., 2016; Luepke et al., 2017). These bacteriophages (or phages) infect and promote bacterial lysis *via* a multi-step process of replication. As these bacterial viruses are specific to bacteria, no activity has been reported against animal or plant cells. Similar to all viruses, phages are metabolically inert in its extracellular form, and they are ubiquitous (Huff et al., 2005).

Various scientific reports suggest that most of the animal viruses and their components are the potent activators of innate as well as acquired immune responses resulting in an increased cytokine, chemokine, reactive oxygen species (ROS) production in humans and animals. These immune responses are mostly due to the viral proteins that stimulate the pro/anti-inflammatory cytokines and ROS production by immune cells (Thannickal and Fanburg, 2000). Some viral proteins such as glycoprotein gp350 and latent membrane protein 1 (LMP-1) from Epstein-Barr virus, showed strong immune expression and also maintains their pro-inflammatory activity by increasing production of interleukin-1beta (IL-1β), tumour necrosis factor-alpha (TNF-1α), IL-6, IL-10 or IL-8 (Mogensen and Paludan, 2001). Similarly, avian influenza A (H5N1) causing severe respiratory disease in humans reported with immune response by increasing inflammatory cytokine and chemokine production (de Jong et al., 2006; Lam et al., 2011).

The efficacy of phage therapy has been proved through pre-clinical and clinical studies administered orally or parenterally (Capparelli et al., 2007; Mann, 2008; Debarbieux et al., 2010; Gavel et al., 2019; Gupta et al., 2019; Nath et al., 2019; Patel et al., 2019). Phages are protein in nature that might induce immunological response as well as induce non-immunological adverse/toxic effects, as mentioned above in the mammalian hosts. Currently, substantial interest has emerged in the field of bacteriophage therapy to be used as anti-bacterial agents. Phages may be introduced to the human body through oral and parenteral routes. The oral route is primarily supposed to eradicate the implicated pathogens present in the gut. Further, if the bacterial pathogens colonizing the gut causing intestinal or extra-intestinal diseases such as diarrhea, dysentery, food poisoning, typhoid, acid peptic diseases, obesity, auto-brewery syndrome, non-alcoholic fatty liver disease, ulcerative colitis, irritable bowel syndrome, other autoimmune disorders etc., if identified in future can be eradicated through oral bacteriophages (Morgan et al., 2012; Rajpal & Brown, 2013; Kishor et al., 2016; Chaturvedi and Nath, 2018; Ganeshan and Hosseinidoust, 2019; Rouse et al., 2020). But, the questions are that: 1) Is oral bacteriophage therapy safe to human health? 2) Are the bacteriophages able to induce adverse immunological responses? If yes, it is only a small dosage or larger dosages cause adverse effects or immunological responses.

Reports on non-immunological and immunological adverse impacts of oral bacteriophages are scarce and yet to be documented especially if high dosages are used for a long duration (Górski et al., 2006; Górski and Weber-Dabrowska, 2005; Górski et al., 2012). Therefore, the present study, was planned to explore the adverse effect of short- and long-term oral administration of high dosages of bacteriophage on rats.

## Materials and Methods

### Chemicals and Reagents

Phosphate buffer saline (PBS, molecular biological grade) was purchased from Sigma-Aldrich (St. Louis, MO). Chloroform and magnesium sulphate were procured from Merck, India. Müller-Hinton agar (MHA), Polyethylene glycol (PEG), agar powder (bacteriological grade), and Tris-hydrochloride AR were obtained from HiMedia Laboratories Pvt. Ltd. India. Sodium chloride laboratory-grade was procured from S D Fine-Chem Limited, India. Gelatin was purchased from BDH Laboratory, Glaxo Laboratories India Limited. All other chemicals used in the present study were of analytical grade available in India.

### Laboratory Animals

A total number of 18 healthy male and female inbred Charles-Foster albino rats (180–220 g) were used in the experiment. All the animals were procured from the Central Animal House (Reg.no.542/02/ab/CPCSEA), Institute of Medical Sciences, Banaras Hindu University, Varanasi, India. All the animals during the experiment were given standard rodent diet procured from M/s. Golden feeds, Mehrauli, New Delhi, India. All the healthy pathogen-free animals were housed in polypropylene cages in the departmental animal house of Microbiology. Food and water were provided *ad libitum*. The rats were kept at a controlled temperature of 22 ± 3°C; humidity of 40–56% and light and dark cycles of 12 h each for one week before and during the experiments. Animal experimental manipulations and postoperative care were conducted according to the Institute for Laboratory Animal Research, US guidelines for the Care and Use of Laboratory Animals. Animals were anesthetized with pentobarbitone (35 mg/kg body weight) intraperitoneally at the end of the experiment for collection of blood through retro-orbital veins. The animals were acclimatized for 5 days before the experiment, and each rat was accessed once daily for clinical signs, behavior, morbidity and mortality. All the animals were allowed to breathe spontaneously during the surgery.

### Bacterial Strain, Isolation, and Identification of *Klebsiella pneumoniae*

A clinical strain of *Klebsiella pneumoniae* was isolated and collected from the patients admitted to the intensive care unit of a tertiary level university hospital of Banaras Hindu University. Mueller Hinton Agar media was used for isolation of the bacteria. The isolated bacteria were confirmed on the basis of colony morphology, Gram staining, biochemical, and molecular technique using *K. pneumoniae* specific primers, i.e., KP16 F′ GCA​AGT​CGA​GCG​GTA​GCA​CAG (nucleotide position 50–70) and KP16 R′ CAG​TGT​GGC​TGG​TCA​TCC​TCT​C (nucleotide position 279–309) with 260 bp product. The PCR cycle used for amplification was 95°C for 3 min followed by 28 cycles of 95°C for 45 s, 58°C for 45 s, 72°C for 1 min, and a final extension at 72°C for 5 min. Antimicrobial susceptibility test (AST) of *K. pneumoniae* was done by using the standard Bauer-Kirby disc diffusion method. The size of inhibition zones was recorded and interpreted according to the Clinical and Laboratory Standards Institute breakpoint Guidelines (CLSI guideline 2018). On antibiotic sensitivity evaluation, the strain was found to be an extensively drug-resistant (XDR). The strain was tested for its susceptibility to gentamicin (GEN, 10 µg), amikacin (AK, 30 µg), netilmicin-sulphate (NET, 30 µg), carbenicillin (CB, 100 µg), piperacillin/tazobactam (PTZ, 100/10 µg), ceftriaxone (CTR, 30 µg), ceftazidime (CAZ, 30 µg), cefepime (CPM, 30 µg), imipenem (IPM, 10 µg), meropenem (MRP, 10 µg), ertapenem (ETP, 10 µg), ciprofloxacin (CIP, 5 µg), levofloxacin (LE, 5 µg), ofloxacin (OF, 5 µg), co-trimoxazole (COT, 25 µg), chloramphenicol (C, 30 µg), fosfomycin (FO 200 µg) and azithromycin (AZM, 15 µg). The sensitivity for colistin and polymyxin was tested by broth dilution technique.

### Source, Sample Collection, and Processing of Water Samples

The water samples were collected aseptically from different water sources (river, ponds, and sewer). One liter volume of water was collected in the sterile bottle from one foot below the surface. Further, the samples were immediately transferred to the laboratory and were processed as per the method described by Gupta et al. (2016) with slight modifications. Before treatment with chloroform, the samples were centrifuged for 10778 × g for 10 min in a refrigerated centrifuge (Remi CPR-24 plus).

### Isolation and Purification of Specific Bacteriophages

Bacteriophage isolation was performed using double agar overlay method with slight modification against this strain from different water sources (river, ponds, and sewer) (Gupta et al., 2016). Bacterial lawn culture (10^8^ CFU/ml suspensions) was made and was incubated for 2 h. Water specimens from different water bodies were treated with 1% chloroform (*v/v*) for 20 min and centrifuged for 10 min at 10778 × *g*, which was dropped over the bacterial lawn and the plates were incubated for overnight at 37˚C. Next day the bacteriolytic activity was noticed in the lawn. Bacteriophages were harvested from the plate using ∼3 ml TMG (Tris-HCl, magnesium sulphate, gelatin pH 7.4) buffer and centrifuged at 10778 × *g* for 15 min. The supernatant (1 ml) was transferred to a 1.5 ml micro-centrifuge tube. Soft agar overlay method was used to get isolated plaques. The process of the soft agar overlay method was repeated till the uniform size and shape of the plaques were observed.

For increasing the number of the bacteriophage, a single plaque was picked up in 1 ml of TMG buffer. The lawn culture of the *K. pneumoniae* was prepared on MH agar and incubated for 4 h to have the bacteria in log phage. The harvested plaque suspension was poured on the whole Petri plate (90 MM) and incubated overnight at 37˚C. The cleared lawn was again harvested in 3 ml of TMG buffer. The Roux bottle containing MH agar was seeded with the host bacteria and brought to the log phase as described earlier. The 3 ml phage harvest was flooded over this lawn and incubated overnight. Next day about 15 ml of TMG was used to harvest the phage was inoculated on six Roux bottle with log phage lawn of the bacterium. After washing each of the Roux bottle yield, the harvest was treated with 1% chloroform for 10 min to lyse the intact bacteria. Each of the six harvests in separate Falcon tube was subjected to centrifugation at 10778 × *g* for 15 min. The supernatant was collected from each of the tubes and subjected to membrane dialysis. The supernatant was loaded in membrane dialysis bags and suspended in a solution containing 25% PEG-8000 and 2.5 M NaCl solution in a big flask at 4˚C for overnight. Two more washing of the phage suspension in the same bag was done by adding fresh PBS (pH 7.2) to the dialysis membrane tube and 25% PEG-8000 and 2.5 M NaCl solution in the outer container. After the third dialysis, all the six thick phage suspension from the dialysis bag was harvested with 1 ml volume/tube in one membrane bag and made up to 15 ml with PBS and again dialyzed with 25% PEG-8000 and 2.5 M NaCl solution overnight at 4˚C. The thick yellowish colour fluid was harvested with 6 ml of TMG. The plaque counting was carried out by using the soft agar overlay method (Kropinski et al., 2009; Mishra and Nath, 2020; Patel et al., 2019). The above *in-house* method gave the yield of about 10^25^ PFU/ml, which was diluted further to achieve 10^20^ and 10^15^ PFU/ml concentration of the bacteriophage.

The endotoxin level of the harvested phage preparations was determined by using Thermo Scientific™ Pierce™ LAL Chromogenic Endotoxin Quantitation Kit ELISA based kit, according to the manufacturer’s instructions. Before performing the test, phage samples and standards of the kit were diluted and were incubated as per instructions. Finally, the color signal was measured using spectrophotometer absorbance at 405–410 nm on a plate reader. The readings were relatively calculated for the presence of endotoxins and defined as the endotoxin content per phage titer (EU/PFU) (Szermer-Olearnik and Boratyński, 2015).

### Experimental Procedure and Acute Toxicity Study (OECD, 2001) of Isolated Bacteriophages

Charles-Foster albino rats of either sex were randomly divided into three groups of six animals (with the equal number of both male and female) in each group, which were fasted overnight. Acute toxicity study was performed as per the Organization for Economic Co-Operation and Development (OECD 423) guideline (Botham, 2002). The control (group 1) received TMG (Tris-HCl, magnesium sulphate, gelatin pH 7.4) buffer and served as a vehicle control group. The experimental groups two and three received a medium (10^15^/ml) and high (10^20^/ml) oral doses of pure bacteriophages, respectively. Animals were observed closely for first 4 h, for any adverse manifestation, like increased motor activity, salivation, convulsion, coma, and death. Subsequent observations were made at regular intervals for 24–48 h. The animals were under further investigation for 2 weeks, while the number of animals died during this phase was noted.

### Sub-Acute Toxicity Study (OECD, 1998) of Isolated Bacteriophages

Charles-Foster albino rats of either sex (equal number of both sexes), weighing between 180 and 220 g were divided into three groups. Group one, two, and three received TMG (Tris-HCl, magnesium sulphate, gelatin pH 7.4) buffer, medium phage concentration (10^15^/ml) and high phage concentration (10^20^/ml), respectively. The doses were administered orally once daily by oral gavage in the volume of 10 ml/kg bodyweight for 28 consecutive days according to the OECD test guideline 407 (Institóris et al., 1998). During the treatment period, animals were observed daily for general behaviour, body weight, food and water intake, hematological profile, liver (total protein, albumin, globulin, total bilirubin, alkaline phosphatase, SGOT, and SGPT) and renal (urea and creatinine) function tests. The weight of all the major organs like liver, kidney, testes/ovaries and adrenal glands was recorded at the end of 28 days of treatment. Histology of all the major organs such as liver, lungs, kidney, heart, spleen, stomach, testes/ovaries, adrenal, and pancreas was also carried out to study any cellular changes after bacteriophage therapy.

### Estimation of Hematological and Biochemical Parameters

At the end of the experiment, blood was collected from the retrobulbar plexus and cardiac puncture using heparinized and non-heparinized capillary tubes. Blood samples in the non-heparinized capillary tube were kept in plain red vials to collect serum, which was further stored for biochemical analysis. However, the heparinized tube’s blood was directly subjected to the estimation of various hematological parameters using a standard instrument. The various hematological parameters such as hemoglobin (Hb), red blood corpuscle (RBC), packed cell volume (PCV), mean corpuscular volume (MCV), mean corpuscular hemoglobin (MCH), mean corpuscular hemoglobin concentration (MCHC), platelets, total leukocyte count and differential leukocyte count were analyzed with blood samples among all the groups. In addition, samples were also subjected to biochemical estimation for the level of magnesium, blood urea nitrogen (BUN), creatinine, uric acid, calcium, phosphorus, potassium, sodium, chloride ion concentration, aspartate transaminase (AST), alanine transaminase (ALT), alkaline phosphate (ALP), creatinine, blood glucose, total protein, and total cholesterol and bilirubin analysis in serum sample using Hematology analyzer (Abbott Model-CD-3700).

### Estimation of Pro-and Anti-Inflammatory Cytokines

The levels of pro and anti-inflammatory cytokines were estimated in all the animals at the end of the experiment in each group, using ELISA assay. Interleukin-1 beta (IL-1β), IL-4, IL-6, and INF-gamma were tested from serum/plasma using standard ELISA assay procedure described by the manufacturer. In brief, ∼50 μl of respective assay diluent was added to each well as per the specific kit standards in different concentrations and samples were pipetted into the wells followed by incubation for 90 min at 37°C. After washing away any unbound substances for a total of five times, the biotin-labelled antibody was added and incubated for at 37°C for 60 min. Further, after washing, the HRP-Streptavidin conjugate working solution was added and incubated at 37°C for 30 min. After washing, TMB substrate was added in all the wells and incubated at 37°C for 15–30 min. After incubation, the reaction was stopped by adding respective stop solution in each well. Immediately after addition of stop solution, optical density (O.D.) was observed at 450 nm in a microtiter plate using Multiskan™ FC Microplate Photometer (Thermo Scientific™, United States). The detailed procedures for calculation of respective cytokines concentration with respect to standards were followed as per the manufacturer’s instructions (Immunotag™ ELISA Kits).

### Measurement of Relative Organ Weight and Histopathological Examination

At the end of the experiment, rats were dissected, and the whole liver, lungs, kidney, heart, spleen, stomach, testes/ovaries, adrenal, and pancreas were excised, freed of fat, blotted dry with clean tissue paper, and then weighed. The organ to body weight ratio was estimated by comparing the weight of each organ with the final body weight of each rat. All the defined samples were placed in 10% neutral buffered formalin for histopathological examination as per standard protocol followed by tissue embedded in paraffin sections, stained with hematoxylin and eosin, and were examined histological changes. Two slides were prepared with 3–6 µM thick tissue sections from all the blocks. One slide was stained with hematoxylin and eosin stain for routine histopathological examination. All the sections were stained with the help of Automatic Linear Slide Stainer (Medimeas, MSS-AS) with hematoxylin and eosin staining method as per standard protocol. The fixed slides were analyzed under an inverted microscope (Nikon ECLIPSE Ts2).

### Estimation of Body Weight, Water and Food Intake

All the experimental animals were subjected to measurement of body weight and food intake before oral dosing of the bacteriophages daily. Briefly, the measurement of daily feed supply (in gms) and the left-over feed by the following day was recorded, and the difference was taken as the daily feed intake by the animal. The data was noted, and average feed and water intake were computed for every three days of the experimental period.

### Clinical Sign

Abnormal behavior in animals was recorded with the time of onset and disappearance. In case, any animal found in a moribund condition or enduring signs of severe distress was humanely euthanized.

### Statistical Analysis

All the data obtained were presented as the mean ± standard error of the mean (SEM) using Sigma-Plot statistical software (Version 11.0). The comparisons involving more than two groups were performed using one-way analysis of variance (ANOVA) followed by post-hoc analysis by Dunnett’s test. The *p* ≤ 0.05 was considered as statistically significant.

## Results

### Isolation and Characterization of the Bacterial Host Strain

*K. pneumoniae* bacterial strain from the clinical source was isolated and tested for susceptibility to different phages. The clinical isolate was confirmed using the colony morphology (Figure 1A), biochemical test, and molecular method using PCR. Further, the clinical strain was tested against the selected 11 antibiotics of six different classes based on the bacterial spectrum, route of administration and type of activity to isolate the multi-drug resistant and XDR strain. Only the XDR strain was selected for further isolation of bacteriophages. The antibiotics panel was tested against the *K. pneumoniae* strains, and only XDR strain based on the tentative zone of inhibition diameter were selected using the latest 2020 CLSI guidelines. Among the tested antibiotics, only fosfomycin was found to be susceptible in disk diffusion assay with a zone of diameter of 24 mm. Fosfomycin was effective as per CLSI listed zone diameter criteria (susceptible, ≤16 mm; intermediate, 13–15 mm; resistant, ≤12 mm). However, other antibiotics were found to be resistant according to the zone of inhibition range. Majority of the isolates showed resistant to multiple drugs (i.e., resistance to two or more classes of the tested antimicrobials), and these were selected for bacteriophage isolation.

**FIGURE 1:** Representative images of isolation of bacteriophages and XDR *Klebsiella pneumoniae*. **(A)** XDR clinical strain of *Klebsiella pneumoniae*, **(B)** High count of bacteriophage and its activity against *Klebsiella pneumoniae* on MHA plate, **(C)** Cultivation of Phage in Roux bottle, **(D)** Membrane dialysis of bacteriophage.

### Isolation of Bacteriophages

Bacteriophages were isolated as per the standardized protocol described by Nath et al., 2019 (Gupta et al., 2016; Nath et al., 2019), while phage counting was done by soft agar overlay method of Nath et al. (2019). The bacteriophages specificity was tested against isolated XDR *K. pneumoniae* clinical strains using plaque formation by using a soft agar overlay method. The isolated phages specific to *K. pneumoniae* formed small and circular plaques that formed well-demarcated big plaques on the top agar plate. The phages were purified and endotoxin level using Pierce LAL Chromogenic Endotoxin Quantitation Kit and was found to be in the safe range of 0.005–0.01 EU/PFU, which was compared and found to be free from endotoxin. Further, the phage titers were determined using log dilutions of the purified phage lysate, and the resulting range of titers were 2.5 × 10^5^ PFU/ml to 5 × 10^20^ PFU/ml. These media (1 × 10^15^ PFU/ml) and high doses (1 × 10^20^ PFU/ml) of bacteriophages were selected for the acute and sub-acute toxicity assay in an animal model (Figure 1). However, the isolated bacteriophages were also tested against different host in order to check the cross-infection such as *E. coli*, *Enterobacter cloacae*, *Proteus mirabilis*, *Salmonella* Typhi, *Staphylococcus aureus*, *Acinetobacter baumannii*, *Pseudomonas aeruginosa*, *Vibrio cholerae*, *Plesiomonas shigelloides*, and *Shigella dysenteriae*.

### Acute Toxicity Study

#### Observation for Behavioral Changes

All the animals were observed for behavioral changes after oral administration of bacteriophages in respective groups. Animals under medium and high dose of bacteriophages showed behavioral changes such as slow response to external stimuli, motionlessness, prostration, and rapid breathing for 60–120 min after the first oral administration through gavage. This change in behavior might have occurred due to a strange uncomfortable experience by the rats for the first time in their life. This speculation is further supported by the observation that behavioral pattern in all the groups was restored to normal with further dosages up to 28 days. Thus, the no-observed-adverse-effect level (NOAEL) for the oral bacteriophage dose was observed. However, after 14 days (∼2 weeks), no animal displayed any behavioral abnormality like trembling, salivation, hair loss, impairment in food and water intake, body weight, sleep, diarrhoea, breathing, altered water consumption, restlessness, lethargy, postural abnormalities, or in physical appearance such as eye colour, mucous membrane, body weight, skin/fur changes, injury, as compared to the animals of the control group. One rat each died in control as well in high bacteriophage dose group after 4 days of the experiment. However, post mortem examinations revealed no macroscopic lesions in the internal organs.

### Sub-chronic Oral Toxicity of Bacteriophages in Rats

#### General Behavior, Body Weight, Food, Water Intake, and Organ to Body Weight Ratio

Isolated pure bacteriophages at medium and high concentrations were administered orally, which did not induce any visible sign in rats of both sexes. However, no lethality was recorded during the 28 days of oral bacteriophage administration. No difference in general behavior, food, and water intake was observed between the tested groups of rats. The changes in body weight during the experimental period and average daily feed intake are presented in Figure 2.

**FIGURE 2:** **(A)** Body weights analysis **(B)** Average daily feed consumption and **(C)** Water consumption (in ml). G1: Control group animals received TMG (Tris-HCl, magnesium sulfate, gelatin pH 7.4) buffer; G2: Animals received oral administration of the medium dose of bacteriophages (10^15^ PFU/ml); and G3: High oral dose of bacteriophages (10^20^ PFU/ml). All the values are presented as mean ± SEM (*n* = 6). No significant difference could be found among the different groups (*p* > 0.05).

Further, the weight of different organs of the animal was noted to calculate the organ weight ratio. As expected, the animal gained weight with time, but no difference in body weight and organ ratio was noted among the control and the bacteriophage treated groups. Similarly, organ weight data was compared with body weight, which was calculated in terms of percentage values of the organ to body weight. The organ to body weight ratio after the completion of the experimental period is presented in Table 1. No significant change in ratio was observed among the experimental group.

**TABLE 1:** Effect of bacteriophages in sub-chronic toxicity assay for the organ to body weight ratio (in percentage).

Group (G)	Liver	Lungs	Kidney	Heart	Spleen	Pancreas	Testis	Stomach
G1	2.87 ± 0.26	0.65 ± 0.05	1.00 ± 0.09	0.51 ± 0.04	0.26 ± 0.04	0.56 ± 0.07	1.17 ± 0.10	0.62 ± 0.08
G2	2.87 ± 0.34	0.64 ± 0.01	0.97 ± 0.05	0.43 ± 0.02	0.28 ± 0.02	0.49 ± 0.06	1.16 ± 0.12	0.55 ± 0.07
G3	2.76 ± 0.37	0.72 ± 0.03	0.83 ± 0.06	0.44 ± 0.02	0.25 ± 0.02	0.42 ± 0.01	1.06 ± 0.05	0.65 ± 0.01

G: Group; G1: Normal control (TMG); G2: Medium oral dose of bacteriophage (10^15^/ml), and G3: High oral dose of bacteriophage (10^20^/ml); All the values are presented as mean ± SEM (*n* = 6). No significant difference could be found among the different groups (*p* > 0.05).

#### Estimation of Hematological Parameters

The level of RBC, WBC, lymphocytes, monocytes, eosinophils, neutrophils, Hb, PCV, MCV, MCH, MCHC, and platelet count were analyzed in all the test groups (Table 2). The changes were non-significant, which suggested that continued bacteriophage therapy did not cause any changes in the blood profile. The reference range was compared according to Alemán et al., 1998. However, clinical laboratory parameters for rats were also considered in order to compare our data in different groups (Clinical Laboratory Parameters, 2021). In blood profile, levels of different types of leukocytes are considered to be the gross immunological biomarker.

**TABLE 2:** Evaluation of hematological parameters assessed after treatment with the bacteriophages in Charles Foster rats.

Parameters	Experimental treatment groups			
	G1	G2	G3	Normal Ref. Range Alemán et al., 1998
RBC (x10^6^/µl)	9.70 ± 0.12	9.34 ± 0.12	8.94 ± 0.14	7.27–9.65
WBC (x10^3^/µl)	4.91 ± 1.21	4.51 ± 1.86	4.98 ± 2.20	1.96–8.25
Lymphocytes (x10^3^/µl)	7.13 ± 0.52	6.00 ± 0.45	7.99 ± 0.31	1.41–7.11
Monocyte (x10^3^/µl)	0.40 ± 0.04	0.51 ± 0.09	0.63 ± 0.14	0.03–0.18
Eosinophils (x10^3^/µl)	0.15 ± 0.00	0.16 ± 0.00	0.17 ± 0.03	0.01–0.16
Neutrophils (x10^3^/µl)	1.42 ± 0.19	1.06 ± 0.02	2.50 ± 0.45	0.22–1.57
Hb (gm/dl)	16.75 ± 0.41	16.75 ± 0.41	16.75 ± 0.41	13–18
PCV (%)	39.18 ± 0.47	39.18 ± 0.47	39.18 ± 0.47	34–42
MCV (fl)	54.90 ± 1.78	54.90 ± 1.78	54.90 ± 1.78	48.5–55.0
MCH (pg)	17.13 ± 0.28	17.13 ± 0.28	17.13 ± 0.28	17.5–22.0
MCHC (gm/dl)	31.73 ± 0.42	31.73 ± 0.42	31.73 ± 0.42	32.0–43.0
Platelet count (thousand/mm^3^)	682.25 ± 12.49	682.25 ± 12.49	682.25 ± 12.49	450–750

G1: Normal control (TMG); G2: A medium oral dose of bacteriophage (10^15^ PFU/ml), and G3: High oral dose of bacteriophage (10^20^ PFU/ml). All the values are presented as mean ± SEM (*n* = 6). No significant difference could be found among the different groups (*p* > 0.05). The normal reference ranges of hematological parameters were mentioned and compared as per animal Clinical Laboratory Parameters.

#### Estimation of Biochemical Parameters

Biochemical parameters of all the animals were evaluated and compared to the healthy control group (Table 3). The biochemical parameters estimated were glucose, total cholesterol (TC), triglycerides (TG), high-density lipoprotein (HDL), low-density lipoprotein (LDL), very-low-density lipoprotein (VLDL), TB (total bilirubin), SGOT, SGPT, ALP, CK-MB, total protein (TP), albumin, globulin, A/G ratio, creatinine, uric acid, blood urea, minerals, and important salts were also analyzed in all the three groups after the end of the study period. Hepatic, renal, lipid, and cardiac biomarkers analysis showed that oral bacteriophage using medium and high doses for 28 days did not alter the blood biochemistry.

**TABLE 3:** Effect of treatment with the bacteriophages on the level of serum biochemical analysis in Charles foster rats.

Parameters	Experimental treatment groups			
	G1	G2	G3	Normal Ref. Range Alemán et al. (1998)
TB (mg/dl)	0.14 ± 0.02	0.09 ± 0.02	0.12 ± 0.01	0.05–0.15
SGOT (U/L)	146.88 ± 8.75	180.90 ± 12.26	186.43 ± 21.10	150–190
SGPT (U/L)	53.13 ± 8.13	37.38 ± 1.21	43.37 ± 11.66	60–90
ALP (U/L)	164.25 ± 24.09	159.59 ± 11.76	148.39 ± 13.16	62–230
CK-MB (U/L)	185.00 ± 26.89	226.40 ± 18.19	209.75 ± 21.88	162–1184
TP (g/dl)	6.21 ± 0.05	7.11 ± 0.33	8.13 ± 0.91	5.2–7.1
A (g/dl)	2.70 ± 0.39	3.78 ± 0.15	3.91 ± 0.32	3.4–4.8
G (g/dl)	2.96 ± 0.04	3.05 ± 0.02	2.57 ± 0.02	1.5–2.5
A/G ratio	1.10 ± 0.02	1.10 ± 0.02	1.26 ± 0.02	1.58–2.67
Creatinine (mg/dl)	0.58 ± 0.10	0.68 ± 0.02	0.64 ± 0.02	0.2–0.5
Uric acid (mg/dl)	0.81 ± 0.06	0.98 ± 0.04	1.21 ± 0.08	0.5–1.4
Blood urea (mg/dl)	29.53 ± 2.55	40.40 ± 3.17	34.90 ± 3.64	12.3–24.6
Calcium (mg/dl)	9.76 ± 0.37	10.51 ± 0.07	11.64 ± 0.18	9.5–11.5
Phosphorus (mg/dl)	6.71 ± 0.58	7.85 ± 0.65	7.79 ± 0.76	5.58–10.41
Na+ (mmol/L)	137.95 ± 2.99	134.68 ± 4.06	130.70 ± 10.30	142–151
K+ (mmol/L)	7.67 ± 1.61	6.15 ± 0.53	5.61 ± 0.69	3.82–5.55
Cl- (mmol/L)	99.95 ± 5.54	96.68 ± 2.37	91.05 ± 2.30	90–106
Glucose (mg/dl)	111.25 ± 5.48	149.48 ± 8.56	152.62 ± 18.38	70–208
TC (mg/dl)	88.52 ± 5.34	117.46 ± 6.75	110.17 ± 5.43	37–85
Triglyceride (mg/dl)	97.38 ± 7.54	109.08 ± 10.13	118.56 ± 14.70	20–120
HDL (mg/dl)	65.17 ± 2.84	73.11 ± 5.11	77.21 ± 1.79	55–80
LDL (mg/dl)	15.39 ± 1.88	14.16 ± 1.03	22.69 ± 1.34	15–24
VLDL (mg/dl)	24.50 ± 3.57	28.00 ± 7.05	25.00 ± 3.32	18–28

G: Group; G1: Normal control (TMG); G2: Medium oral dose of bacteriophage (10^15^/ml), and G3: High oral dose of bacteriophage (10^20^/ml); No significant difference could be found among the different groups (*p* < 0.005). All the values are presented as mean ± SEM (*n* = 6). No significant difference could be found among the different groups (*p* > 0.05). The normal reference ranges of serum biochemical parameters were mentioned and compared as per animal Clinical Laboratory Parameters.

#### Estimation of Cytokines Level

Interlukin-1 beta (IL-1β), IL-4, IL-6, and INF-gamma levels were estimated in all the animals and the test was performed using ELISA assay. The results of all the cytokines were compiled and graphically presented in Figure 3. The control group showed cytokine values of IL-4, IL-1β, IL-6, and INF-gamma as 109.00 ± 11.72, 76.21 ± 17.45, 84.00 ± 11.72, and 53.33 ± 13.74 pg/ml, respectively. The cytokines assay results showed that pro-and anti-inflammatory level of cytokines varied but without statistically significant difference.

**FIGURE 3:** Experimental animals were fed with bacteriophages for 28 days, and the serum was subjected for the estimation group of pro- and anti-inflammatory cytokines using ELISA assay **(A)** IL-4, **(B)** IL-6, **(C)** IL-1beta, and **(D)** INF-gamma. The experimental values were performed in triplicate, using blood samples from three independent animals. G1: Control group animals received TMG (Tris-HCl, magnesium sulfate, gelatin pH 7.4) buffer, G2: Animals received oral administration of a medium dose of bacteriophages (10^15^/ml), and G3: High oral dose of bacteriophages (10^20^/ml). All the values are presented as mean ± SEM (*n* = 6). No significant difference could be found among the different groups (*p* > 0.05).

#### Histopathological Analysis

After the end of the experiment, tissue samples were collected, which were fixed and stained in order to examine any histopathological changes in all major organs. The changes were compiled using microscopic images as seen in Figure 4 and Table 4. The results depicted no notable significant changes in the GIT as well as other major organs as determined by a pathologist. Thus, no significant histopathological changes were observed in collected tissues after the experimental period suggesting safe bacteriophage therapy.

**FIGURE 4:** Histopathological observation of major tissues obtained from GIT and other major organs of Charles Foster rats fed with (G1) vehicle control, (G2) medium-dose bacteriophages (1 × 10^15^ PFU/ml), and (G3) high dose of bacteriophages (1 × 10^20^ PFU/ml). Experimental animals were fed with phages for 28 days and were sacrificed. All the isolated tissues were fixed and stained with hematoxylin-eosin and observed under a microscope.

**TABLE 4:** Summary of histopathology findings (H and E stain).

Organ	Finding	G1A1	G1A4	G2A1	G2A4	G3A1	G3A4
**Lungs**	Mononuclear cell infiltration, multifocal	0	1	1	0	1	0
	Bronchitis, no alveolar lymph	0	0	0	0	0	0
	Normal and some enlarged alveoli, bronchopneumonia, multifocal	0	0	0	0	0	0
**Heart**	No abnormality detected	0	0	0	0	0	0
**Adrenals**	Accessory cortical nodule, focal, unilateral	0	0	0	0	0	0
	Cortical vacuolation, diffuse, bilateral	0	0	0	0	0	0
**Eyes**	No abnormality detected	0	0	0	0	0	0
**Liver**	Mononuclear cell infiltration, focal	0	1	0	0	0	1
	Hepatocellular vacuolation, diffuse	0	0	0	0	0	0
**Spleen**	No abnormality detected	0	0	0	0	0	0
**Thymus**	No abnormality detected	0	0	0	0	0	0
**Kidneys**	Basophilic tubule, focal	0	0	0	0	1	0
	Mononuclear cell infiltration, multifocal	0	0	0	0	0	0
**Testes**	Tubular degeneration, multi focal, bilateral	0	1	0	0	0	0
	Tubular degeneration, focal, unilateral	0	0	0	0	0	0
**Stomach**	Normal gastric mucosa, no necrosis	0	1	0	0	0	0
**Duodenum**	No abnormality detected	0	0	1	0	0	0
**Jejunum**	No abnormality detected	0	0	0	0	0	0
**Ileum**	No abnormality detected	0	0	0	0	0	0
**Caecum**	Neutrophilic infiltration, diffuse	0	0	0	0	0	0
**Colon**	Neutrophilic infiltration, diffuse	0	0	0	0	0	0
**Rectum**	Neutrophilic infiltration, diffuse	0	0	0	0	0	0
**Pancreas**	No abnormality detected, normal tissue	0	0	0	0	0	0

## Discussion

In the present study, we decided to explore the possibility of using oral bacteriophages at high concentration for many weeks to see the adverse/toxic and immunological effects in a rodent model. We divided adult Charles Foster rats into three groups: A group without intervention and two experimental groups given phage dosages of 10^15^ PFU/ml and 10^20^ PFU/ml daily for 28 days. Various parameters like behavioral changes, body weight, food and water intake, and organ to body weight ratio, hematological, biochemical, cytokines levels and histopathological changes were examined. It was intriguing to see that there were no significant changes in any of the parameters mentioned above as compared to the control group. Both the groups of rats with the medium and high dosages of phages exhibited a similar kind of response. The behavioural changes observed during the first 2 h might be due to discomfort and strange experience due to gavage procedure. This speculation is further proved as no such response could be noted during subsequent bacteriophage dosages given in the same way. The absence of lethality after phage administration indicates that oral phage therapy is safe and free of toxicity. Sulakvelidze et al. (2001) also have observed that doses between 10^5^ and 10^11^ through oral, rectal, topical and respiratory routes did not cause a visible adverse effect. When Bogovazova et al. (1991) and Bogovazova et al. (1992) administered bacteriophage specific to *Klebsiella spp*. through intramuscular, intraperitoneal and intravenous in rats and guinea pigs to study the pharmacokinetics and toxicology of the phages, no acute toxicity, macroscopic or microscopic changes could be noticed (Bogovazova et al., 1991; Bogovazova et al., 1992). The observation was made even though the doses given were 3500 times higher than those projected for humans. In the continuation, this group performed another study and demonstrated that human patients infected with *Klebsiella spp*. given specific bacteriophage were not associated with any toxicity.

It is interesting to see that the total and differential leukocyte counts remain unaffected indicating absence of induction of inflammatory response against the fed bacteriophages. It is intriguing to see that pro-inflammatory (IL-1β, IL4, and IL6) cytokines were not altered despite such a high dose of bacteriophage (Górski et al., 2012; Hong et al., 2016; Van Belleghem et al., 2018). IL4 leading to suppression of TH1 response could also be negated as no significant change was be seen. IFNγ is also known as type II interferon that has a critical role both in innate and adaptive immunity against viral, some bacterial and protozoal infections. IFNγ is known to inhibit viral replication directly. The indifference in the levels of IFNγ in the experimental group than the control group suggests that bacteriophages given orally failed to induce the overproduction of IFNγ. The scientific data suggested that any form of the pathogen should initiate the first immune response as inflammation (Belkaid and Hand, 2014). Sensitized cells result in the production and release of pro-inflammatory cytokines, which helps the immune system to repel the incoming pathogens such as pathogenic bacteria and viruses (Ganesh et al., 2013; McCarthy et al., 2013). In support of the present study, the earlier report states a minimal alteration in the serum cytokine levels when T4 bacteriophages were administered orally (Miernikiewicz et al., 2013). Hong *et al.* have shown that at times phage treated rats had lower cytokine level as compared to controls (Hong et al., 2016). Thus, therapeutic feeding of bacteriophages targeting any gut bacterial pathogen implicated induces either minimal or no adverse effect. Even though oral administration of phages was given for 4 weeks, it did not cause a significant immunological response. The possible explanations for this observation may those phages are the part of normal microbiota/virobiota of humans and therefore not eliciting the significant detrimental immune responses. In support of the above statement there are many reports suggesting that the phages may be the part of human microbiota (Minot et al., 2011; Navarro and Muniesa, 2017; and; Van Belleghem et al., 2019). It was also found that against T-like bacteriophages, natural antibodies may be presented due to it’s natural existence as a part of normal flora (Dabrowska et al., 2014). Łusiak-Szelachowska et al., 2014 has reported minimal altered immune response as the outcome of the phage therapy was not affected by the appearance of neutralizing antibodies. However, exact mechanism of anti-phage cellular response is yet to be demonstrated. The other possibility is that high oral bacteriophages might cause desensitization or immune paralysis resulting in all the immunological parameters in normal range. If this is the case, this immune paralysis phenomenon will be quite useful in cases where prolong bacteriophage therapy is warranted.

Therefore, it seems that oral bacteriophage therapy is safe, and it can be used to eradicate the specific pathogen present in the gut. However, it would have been better if the effect of oral phage therapy on alteration of gut microbiota was also evaluated. Further, one must study to explore whether phage genes/genome is getting integrated into the genome of host bacteria or other related bacteria to convince the regulatory authority. The literature available in this field is still scarce and contradictory, and there is a need to make desperate attempts to make more in-depth investigations.

## Conclusion

Thus, in the conclusion of the above-detailed toxicity and immunobiological activity of medium and high oral administration of bacteriophages of XDR *Klebsiella pneumoniae*, the therapeutic feeding of bacteriophages suggesting no adverse effect was found when animals were challenged at high PFU count (1 × 10^20^/ml). Continued phage therapy for 28 days was found to be safe with respect to animal hematology, biochemistry, body weight, feed intake, histopathology, and vital behavioral parameters. Besides, the immunological response of the animal after the experimental period was found safe with minimal change in pro and anti-inflammatory level of cytokines, indicating that the oral administration of bacteriophages would appear to be a safe practice for fighting against XDR or any other bacterial pathogens and no adverse acute immune response was noted during the study period.

## Data Availability

The original contributions presented in the study are included in the article/Supplementary Material, further inquiries can be directed to the corresponding author.
